The article "Living with Yourself: Innate Lymphoid Cell Immunometabolism" was retracted in 2022. Reason: duplicate publication.

# Living with Yourself: Innate Lymphoid Cell Immunometabolism

**DOI:** 10.3390/cells9020334

**Published:** 2020-02-01

**Authors:** Marion Rolot, Timothy E. O’Sullivan

**Affiliations:** Department of Microbiology, Immunology, and Molecular Genetics, David Geffen School of Medicine at UCLA, Los Angeles, CA 900953, USA; rolotmarion@gmail.com

**Keywords:** innate lymphoid cells, immunometabolism, obesity, microbiota, diet

## Abstract

Innate lymphoid cells (ILCs) are tissue-resident sentinels of the immune system that function to protect local tissue microenvironments against pathogens and maintain homeostasis. However, because ILCs are sensitively tuned to perturbations within tissues, they can also contribute to host pathology when critical activating signals become dysregulated. Recent work has demonstrated that the crosstalk between ILCs and their environment has a significant impact on host metabolism in health and disease. In this review, we summarize studies that support evidence for the ability of ILCs to influence tissue and systemic metabolism, as well as how ILCs can be regulated by environmental changes in systemic host metabolism. We also highlight studies demonstrating how ILC- intrinsic metabolism influences their activation, proliferation, and homeostasis. Finally, this review discusses the challenges and open questions in the rapidly expanding field of ILCs and immunometabolism.

## 1. Introduction

Innate lymphoid cells (ILCs) consist of a heterogeneous family of lymphocytes that do not express rearranged antigen receptors, but instead express a wide variety of germline-encoded activating and inhibitory receptors [1,2]. ILCs can be identified in lymphoid and non-lymphoid tissues, and are enriched at epithelial barrier surfaces such as the intestine, lung, and skin [1,2]. Recent evidence has suggested that mature ILCs can be further classified into group 1, 2, and 3 ILCs based on different expression of transcription factors, cell surface markers, and effector cytokines [1,2]. Group 1 ILCs, which include natural killer (NK) cells and ILC1s, can be distinguished from other ILCs based on their constitutive expression of the transcription factor T-bet, co-expression of activating receptors NKp46 and NK1.1, and production of interferon (IFN)-γ following stimulation with proinflammatory cytokines interleukin (IL)-12 and IL-18 [3]. NK cells, the original member of group 1 ILCs [4], are cytotoxic innate lymphocytes that constitutively express the transcription factor Eomes and the integrin CD49b (also known as DX5 or α_2_β_1_ integrin), and survey peripheral tissues by constant circulation through the vasculature to perform host immunosurveillance against viruses and tumors [5,6,7,8]. In contrast to NK cells, ILC1s lack Eomes and CD49b expression, but express the inhibitory receptor CD200R [9]. ILC1s are long-term tissue resident in peripheral organs, and may be required to protect the host from bacterial infections at barrier sites such as the intestine [5,6,10,11,12,13,14]. Group 2 ILCs, which consist of ILC2, express the transcription factor GATA3 and produce type 2 cytokines such as IL-4, IL-5, and IL-13, along with the tissue reparative factor amphiregulin, to promote host resistance to helminth infection [15,16,17,18,19]. Lastly, group 3 ILCs consist of lymphoid tissue inducer (LTi) cells and NKp46^−^ and NKp46^+^ ILC3s that express retinoid-related orphan receptor γt (RORγt) and can produce IL-22, Il-17A, and lymphotoxin to maintain tissue homeostasis and antibacterial immunity in the intestine [20,21,22,23,24,25].

ILCs are rapid producers of both proinflammatory and regulatory cytokines in response to local injury, inflammation, pathogen infection, or commensal microbiota perturbation [1,2]. Because most ILCs have been shown to be tissue-resident during homeostasis (with the exception of circulating NK cells) in almost all organs analyzed [5,14], their ability to quickly respond to tissue stress and inflammation underpins their critical role in regulating tissue homeostasis and repair during infection or injury [1,2,26]. However, persistent inflammatory signals can also lead to unrestrained activation of certain ILC populations at barrier surfaces, thereby exacerbating colitis, dermatitis, and contributing to tumorigenesis [27,28,29,30,31]. Collectively, these studies demonstrate the impact of ILCs in tissue microenvironments and highlight the delicate balance between ILC-mediated immune protection and pathology. Recent reports have identified certain ILC populations in non-barrier tissues with important host metabolic function (i.e., liver and adipose tissue) and collectively suggest a broader role for ILCs in the maintenance of both tissue homeostasis and systemic host metabolism [32,33]. Given the contribution of ILCs to tissue inflammation in other diseases, it may not be surprising that recent studies have also implicated ILCs in the disruption of host tissue homeostasis and systemic metabolism during diet-induced obesity [14,34,35,36]. This review summarizes recent findings in the field of ILC biology that address three central questions in the field of immunometabolism: What are the cell-intrinsic metabolic pathways that are utilized by ILCs during activation and homeostasis? How does host tissue and systemic metabolism impact the homeostasis or activation state of ILCs? And finally, how do ILCs maintain or disrupt host tissue and systemic metabolism in disease states?

## 2. Cell-Intrinsic Metabolism of ILCs

The study of cellular immunometabolism focuses on cell-intrinsic changes to metabolic pathways that influence discrete cellular states such as activation, proliferation, and homeostasis. Naïve lymphocytes are generally thought to be quiescent and largely use metabolic pathways that efficiently metabolize glucose through glycolysis-linked mitochondrial oxidative phosphorylation (OXPHOS) to generate energy in the form of adenosine triphosphate (ATP). During activation, adaptive and innate immune cells increase the rate of glycolysis to meet higher biosynthetic demand by metabolizing glucose into lactate in a process called aerobic glycolysis to provide the cell with essential precursors for amino acids, lipids, and nucleotides [37,38,39]. However, the metabolic pathways that ILCs utilize during homeostasis and host defense have only recently begun to be unveiled. In this section, we summarize the relatively few studies that offer insight on the cell-intrinsic metabolic pathways used by ILCs during steady state and activation.

### 2.1. Group 1 ILC-Intrinsic Metabolism

Similar to naïve T cells, freshly-isolated naïve mouse and human NK cells rely on OXPHOS (Figure 1A), but quickly shift to aerobic glycolysis following culture with high-dose IL-15, which induces the activation and proliferation of NK and T cells [40,41,42,43,44]. In terms of effector function, NK cells may differ from T cells as the requirement of aerobic glycolysis for optimal IFN-γ production may vary depending on the stimuli inducing NK cell activation. NK cells can utilize an aerobic glycolysis-independent mechanism for IFN-γ production following stimulation with IL-12 and IL-18 ex vivo [40]. By contrast, another study found that IL-15-expanded NK cells require aerobic glycolysis for optimal IFN-γ production following IL-2 and IL-12 stimulation in vitro [41]. However, because in vitro culture conditions may not accurately reflect physiologic levels of oxygen, nutrient concentrations (i.e., glucose, glutamine, and fatty acids), and cytokine concentrations, these conclusions may be limited by how the differences in these conditions impact cellular metabolism in vitro versus in vivo.

Nevertheless, the in vivo role for aerobic glycolysis in promoting NK cell cytokine production remains unclear. IL-15 stimulation in vitro and stimulation with the toll-like receptor-3 ligand polyinosinic-polycytidylic acid (poly(I:C)) in vivo increase mammalian target of rapamycin (mTOR) signaling, which is associated with an increase in aerobic glycolysis in activated NK cells [42]. Poly(I:C) injection and murine cytomegalovirus (MCMV) infection, both of which induce IL-15, IL-12, and IL-18 in vivo [45], lead to decreased IFN-γ production by NK cells in the presence of either glycolysis pathway inhibitors or mTOR inhibitors [41,46], suggesting that pro-inflammatory cytokine induction of mTOR signaling may lead to increased aerobic glycolysis in NK cells to potentiate IFN-γ production. In support of this hypothesis, NK cell cytotoxic function and viral control was shown to depend on mTOR-dependent glycolysis following IL-15 activation in vitro and MCMV infection in vivo. Similarly, inhibition of glycolysis may be responsible for the decreased cytotoxicity of NK cells during immunosurveillance in a Kra*s*-driven lung cancer model [47]. In contrast, IL-15 was found to prime NK cell function in an mTOR- and glycolysis-independent manner because treatment with the IL-15 superagonist ALT-803 can rescue NK cell-dependent control of MCMV in mice treated with glucose metabolism or mTOR pathway inhibitors [48]. However, it remains difficult to determine the intrinsic role of mTOR signaling on NK cell effector function from these previous studies in vivo because systemic treatment with these inhibitors during inflammation could have cell-extrinsic effects that decrease NK cell IFN-γ production. This point is supported by the observation that NK cell-intrinsic loss of mTOR does not impact IFN-γ production during MCMV infection or following ex vivo stimulation with IL-12 and IL-18 [42]. It should be noted, however, that mTOR-deficient NK cells do not progress past at an immature stage, suggesting that mTOR signaling is necessary for the optimal proliferation of immature NK cells to populate the mature NK cell pool during homeostasis [42]. These observations make it difficult to dissociate the role of mTOR-induced IFN-γ production in mature rather than immature NK cells. To rule out these observed developmental defects, adoptive transfer studies using NK cells with inducibly-deleted mTOR suggest that while mTOR is dispensable for mature NK cell homeostasis, its signaling is necessary for optimal NK cell cytotoxicity and proliferation during poly(I:C)-induced inflammation [42]. Therefore, while increased mTOR signaling and aerobic glycolysis can control NK cell proliferation and cytotoxicity in NK cells during inflammation-induced activation (Figure 1B), the metabolic pathways NK cells utilize to produce IFN-γ in vivo remain unclear.

Although the growing consensus is that mTOR inhibition in vivo restrains NK proliferation and cytotoxicity early during inflammation, recent studies have also demonstrated that inhibition of mTOR following periods of inflammation or proliferation can lead to enhanced survival of group 1 ILCs. In those studies, autophagy was enhanced by inhibition of mTOR, limiting apoptosis and promoting survival of ILC1 or NK cells in a cell-intrinsic manner during homeostatic proliferation or viral infection [49,50,51]. Whereas autophagy is critical for the development of all known lymphocytes [51,52], autophagy was not found to be necessary for the basal turnover and homeostasis of mature ILCs and their precursors in a cell-intrinsic manner through inducible deletion of the core autophagosome machinery component *Atg5* [51]. Thus, while initial activation of mTOR signaling is required for optimal proliferation of NK cells in vivo, subsequent metabolic adaptation to suppress anabolic mTOR-induced glycolysis and induce catabolic autophagy is essential to inhibit apoptosis in group 1 innate lymphocytes following periods of cell differentiation or stress, such as homeostatic proliferation or viral infection.

### 2.2. ILC2- and ILC3-Intrinsic Metabolism

Although aerobic glycolysis-fueled proliferation and effector function are key characteristics of NK cell and T cell responses to activating signals in vitro and in vivo, whether other ILC populations utilize similar metabolic pathways to fuel effector responses remains unclear. HIF1α-regulated glycolysis appeared to be important for ILC2 development. Shifting the balance between oxidative phosphorylation and glycolysis towards glycolysis-attenuated ILC2 development and function [53,54]. Recent studies have demonstrated that both ILC2 precursors and mature ILC2s express high levels of the metabolic enzyme arginase-1 [55,56]. Arginase-1 metabolizes the amino acid L-arginine into urea and ornithine to generate downstream metabolites to fuel bioenergetic pathways critical for cellular proliferation [57]. In one study, conditional deletion of arginase-1 in all lymphocyte-lineage cells revealed defects in lung ILC2 proliferative capacity and cytokine secretion during papain-induced lung inflammation in the absence of apparent developmental defects [55]. Reduced proliferation and effector function in lung ILC2s was caused by cell-intrinsic defects in arginine catabolism and aerobic glycolysis [55] (Figure 1C, left panel). Using a genetic method to selectively target mature ILC2s, however, another study found that deletion of arginase-1 did not impact lung ILC2 proliferation or production of IL-5 and IL-13 during helminth infection [56]. These conflicting results suggest either that the requirement of arginase-1 activity to promote effector functions in mature ILC2s may be dictated by specific inflammatory contexts, or that arginase-1 activity may metabolically license ILC2 precursors to potentiate the optimal effector functions of mature ILC2s. While transcriptional profiling of intestinal ILC3s has revealed pathways enriched in glycolysis [58], in line with another study showing mTOR to be required for NCR^+^ ILC3 development [42], arginase-1 was found to be dispensable for ILC3 development and anti-bacterial immunity [55]. Together, these results suggest that ILC3s may not utilize arginase-1 activity to fuel glycolysis and cellular proliferation during development and inflammation. Mouse and human ILC3s have been recently shown to rely on glycolysis, mitochondrial respiratory function, and lipid oxidation (including de novo lipidogenesis) for effector function [59]. Specifically activation of the mTOR-HIF1α pathway and production of mitochondrial reactive oxygen species (mROS) were required for cytokine production and cell proliferation after activation by IL-1β and IL-23 or during *Citrobacter rodentium* infection [59] (Figure 1D).

Other studies suggest that intestinal ILC2s express a genetic signature enriched in genes involved in fatty acid metabolism [60], and intestinal ILC2s as well as ILC3s have been shown to uptake extracellular fatty acids from their environment during homeostasis [61]. Inhibition of systemic fatty acid oxidation (FAO) by treatment of etomoxir in vivo, but not systemic inhibition of glycolysis, reduced intestinal ILC2 accumulation and production of IL-13 and IL-5 in response to helminth infection [61]. These results suggest that ILC2s may be metabolically distinct from other lymphocytes in that they could preferentially use lipid-fueled FAO to support their proliferation and effector functions during pathogen-induced inflammation (Figure 1C, right panel). Indeed, this mechanism may not be specific to intestinal ILC2s because attenuation of FAO in autophagy-deficient lung ILC2s was associated with impaired effector function during in vivo stimulation with IL-33 [54]. Although ILC2s and ILC3s have increased rates of extracellular fatty acid uptake compared to regulatory T cells in the small intestine, blockade of FAO by etomoxir does not perturb ILC2 homeostasis in vivo [61]. Therefore, future work will be needed to uncover the specific metabolic pathways that are utilized by ILC2s and ILC3s during homeostasis.

## 3. Tissue Immunometabolism and ILCs

The study of tissue immunometabolism focuses on how immune cells influence tissue and systemic metabolism in the steady state and in response to environmental changes and has been reviewed in detail previously [33]. Reciprocally, the field also investigates how changes in local and systemic metabolism (often in metabolic disease settings) influence the immune system. Metabolic tissues, such as the liver and adipose tissue, consist of stromal, parenchymal, and immune cells that coordinate their cellular functions to maintain the metabolic functions carried out by parenchymal cells (i.e., hepatocytes and adipocytes). Immune and stromal populations are thought to maintain these functions through the production of various cytokines, growth factors, and hormones [33]. In addition, the immune system has evolved to be closely regulated by host nutritional status and environmental changes [33]. In this section, we will review studies demonstrating how ILCs influence tissue immunometabolism, and how environmental metabolic changes influence ILC biology.

### 3.1. ILCs Maintain Metabolic Homeostasis

The main function of the white adipose tissue (WAT) is to store excess lipids from the circulation when nutrient availability exceeds energy expenditure. In addition, when nutrients are limited, adipocytes induce lipolysis to break down stored lipid droplets to provide lipid fuel to other tissues [62,63]. Adipocytes also produce a plethora of secreted molecules called adipokines (i.e., leptin, resistin, and adiponectin) that maintain local and systemic tissue metabolic homeostasis [33]. A key characteristic of metabolic fitness of the adipose tissue is insulin sensitivity, which has been shown by several studies to be maintained by type 2 immune cells such as alternatively activated macrophages (M2), eosinophils, and Th2 cells [64,65,66,67]. Although the roles of these cells in adipose metabolic homeostasis have been reviewed previously [33,67], ILC2-derived IL-5 and IL-13 has recently been shown to maintain insulin sensitivity in lean mice through the recruitment of eosinophils by IL-5, and by maintenance of M2 macrophage polarization by IL-13 [64,65]. ILC2s may also control certain aspects of weight gain in mice, as IL-33-deficient mice (which have reduced functional ILC2s) develop spontaneous weight gain and fat mass on a low fat diet [68]. However, whether the spontaneous weight gain observed during IL-33 deficiency is caused by deficiencies in adipocyte-intrinsic mitochondrial respiratory capacity and metabolism [69] or ILC2-derived IL-5 production remains unclear.

A recent study demonstrated through lineage tracing and parabiosis experiments that the adipose tissue contains a heterogeneous mixture of group 1 ILCs, consisting of circulating mature NK cells and tissue-resident ILC1s and immature NK cells during steady state [14]. Although these cells do not display activated phenotypes in lean mice, a subsequent study proposed that group 1 ILCs function to maintain macrophage homeostasis in the visceral white adipose tissue (VAT) by preferentially killing adipose M2 macrophages in vivo [36]. This was suggested to be caused by enhanced expression of the NKG2D ligand RAE-1 on adipose macrophages during homeostasis [36]. However, these results are controversial because the consensus in the field is that M2 macrophages serve a protective rather than detrimental role in the homeostasis of the adipose tissue [33,67], and our laboratory, in addition to others, have not observed metabolic defects nor altered M2 macrophage homeostasis in group 1 ILC-deficient mice or NKG2D-deficient lean mice [70]. Therefore, while group 1 ILCs are enriched in the adipose tissue, their role in maintaining adipose macrophage numbers and metabolic fitness during homeostasis will need more precise investigation.

Although gut commensal bacteria are not of host origin, current evidence strongly suggests that the microbiota can influence the host response to dietary intake by altering the metabolism, storage, and absorption of calories [71]. This notion of the microbiota as a metabolic “organ” is highlighted by studies demonstrating that germ-free rats have reduced weight and harvest less energy despite increased food intake compared to microbiota-sufficient controls [72,73]. Emerging evidence suggests that ILC3s can regulate the homeostasis and composition of the intestinal microbiota. In mice, ILC3s are the main source of IL-22 [23,24,74], which is important to stimulate antimicrobial peptides and mucins from intestinal epithelial cells to contain commensal bacteria within the intestine [74,75]. In addition, ILC3s function to promote fucose transfer to the surface of epithelial cells in the intestine, which is used by the commensal microbiota as a carbohydrate source [76], and have been found to be important in controlling cecal homeostasis in a non-redundant manner [77]. Given the intimate relationship between ILC3s and the microbiota, it will be of interest to investigate whether ILC3-mediated control of the microbiota can indirectly regulate whole-body metabolism.

### 3.2. Environmental Changes in Host Metabolism Influence ILC Biology

Although ILCs have been shown to have important roles in the regulation of host metabolism, several studies have also shown that environmental changes to host metabolism can directly regulate key facets of ILC biology. Following exposure to cold temperatures, certain WAT tissues are able to perform thermogenesis to provide heat for the host by inducing beige adipocytes with enhanced expression of uncoupling protein 1 (UCP1). This environmental change in temperature is sensed by adipose-resident ILC2s in response to local production of IL-33 to produce IL-13 and potentiate the lineage commitment and proliferation of PDGRα^+^ stromal cells to beige fat cells [78]. IL-33 can also induce the production of methionine-enkephalin peptides by adipose ILC2s, resulting in increased UCP1 expression in the WAT [68]. While this provides a direct example of environmental metabolic changes resulting in ILC responses, how IL-33 is produced in response to cold stress, and the host cells that produce IL-33 in vivo are unknown.

The intestinal microbiota can also influence ILC homeostasis by providing bacterial-derived metabolites to host cells based on dietary input from the environment. Vegetable-derived phytochemicals can influence ILC3 and ILC2 cytokine secretion and survival by modulation of the transcription factor aryl hydrocarbon receptor (AHR) [79,80,81]. Activation of AHR increases ILC3 function but decreases ILC2 function, influencing the balance of ILC3–ILC2 responses in the gut [82]. The microbiota can also indirectly influence levels of indole 3-aldehyde, a tryptophan-derivative that binds to AHR, to promote IL-22 production by ILC3s [83]. Furthermore, signaling of microbiota-derived short-chain fatty acid (SCFA) via free fatty acid receptor 2 (FFAR2) can induce colonic ILC3 proliferation and production of IL-22 to promote intestinal barrier immunity[84] while ILC2s are inhibited by the SCFA butyrate, leading to improvement of allergic asthma symptoms [85]. ILC3s may be unique in their dependence on microbiota-derived metabolites, because NK and ILC2 development is not perturbed while NKp46^+^ ILC3s can be reduced in germfree mice [25,86,87]. However, other studies have reported that ILC3 development is normal in the absence of the microbiota [22,23,74], suggesting that the development and homeostasis of ILCs may not depend on the microbiota. Instead, oxysterols, synthetized by fibroblastic stromal cells, can induce the migration of ILC3s in colonic lymphoid tissues during development and inflammation [88,89]. Using single cell RNA sequencing analysis of ILC populations in the small intestine, a recent study found a high degree of transcript regulation in ILC1s and ILC2s in response to the presence of commensal microbiota, while transcript levels of IL-22 did not change in ILC3s [58]. These results collectively suggest that the microbiota may influence certain aspects of the steady-state transcriptional landscape rather than development of ILCs in the intestine, although future work is needed to clarify the role of the microbiota on ILC function and development.

Whether or not host microbiota directly influence ILC development and effector function, there is clear consensus in the field that diet can influence ILC biology. It has recently been showed that cyclic effector function of ILC3s and ILC2s was influenced by food intake, independently of circadian cycle. ILC3s respond to food-induced expression of neuropeptide vasoactive intestinal peptide (VIP) allowing them to maintain epithelial barrier integrity [90]. Dietary nutrient deficiencies, such as vitamin A or vitamin D deficiency, leads to a loss of ILC3s in the gut [91,92,93], while ILC2 number and effector function are enhanced by increased FAO and acquisition of long-chain fatty acids [61]. Dietary nutrient oversupply of fat, which leads to obesity, results in the hypertrophy of adipocytes, limiting their nutrient and oxygen availability and resulting in a sustained stress response in both adipocytes and stromal cells [94,95,96]. This stress response results in the recruitment, activation, and proliferation of IFN-γ-producing circulating CD8^+^ T cells, Th1 cells, and NK cells as well as tissue-resident adipose ILC1s to drive the accumulation of proinflammatory macrophages in the adipose tissue [14,34,35,97,98,99]. Together, these studies highlight the sensitive balance between environmental dietary inputs and ILC homeostasis and activation and warrant further investigation into the mechanisms of these processes.

### 3.3. ILC Activation Disrupts Metabolic Homeostasis during Diet-Induced Obesity

During diet-induced obesity, unrestrained type 1 responses promote the production of the cytokines tumor necrosis factor (TNF)-α and IL-6 by proinflammatory macrophages, which can reduce insulin sensitivity over time [100,101,102]. Given that group 1 ILCs are activated during diet-induced obesity in mice, recent studies have shown that systemic depletion of NK1.1^+^ or NKp46^+^ cells reduces diet-induced obesity-associated insulin resistance by decreasing the polarization of proinflammatory macrophages [34,35,103]. Although the genetic or antibody depletion methods utilized in these studies also reduced adipose NKT cells, which can suppress insulin resistance during diet-induced obesity [104,105], adoptive transfer of CD49b^+^ splenic NK cells into the VAT of *Ifng^−/−^* mice was sufficient to exacerbate insulin resistance following high fat diet (HFD) administration [35]. Similarly, adoptive transfer of splenic CD49b^+^ NK cells into *Nfil3^−/−^* mice was sufficient to enhance insulin resistance during diet-induced obesity [34], demonstrating that CD49b^+^ NK cells can contribute to insulin resistance in the presence of an intact adaptive immune system. However, because of the heterogeneity of group 1 ILCs present in the adipose tissue, the contribution of other tissue-resident group 1 ILCs in obesity-associated insulin resistance remained unknown from these studies. Although recent data indicate a protective role of white adipose tissue ILC2s during homeostasis, ILC2s and ILC3s from the small intestine, but not from white adipose tissue, were found to promote weight gain and insulin resistance during diet-induced obesity in mice [106]. These results suggest that the individual roles of tissue-specific and circulating subsets of ILCs need to be taken into account during obesity.

Recent evidence suggests that adipose-resident ILC1s proliferated locally and produced the highest amounts of IFN-γ early during HFD feeding compared to other known IFN-γ producing lymphocytes in the adipose tissue, including NK cells [14]. Furthermore, adipose ILC1s polarized adipose proinflammatory macrophages and contributed to metabolic dysfunction to a greater extent on a per cell basis (relative to immature or mature NK cells), suggesting that adipose ILC1 responses to HFD-induced inflammation are the most potent among group 1 ILCs in driving disease progression [14]. Higher numbers of circulating and adipose ILC1-like cells expressing IFN-γ have also been detected in obese subjects. Numbers of adipose ILC1-like cells are further increased in obese subjects with type 2 diabetes and correlate with insulin resistance [107]. A caveat with this hypothesis is that the genetic ablation tools to definitively differentiate between the contribution of each subset of group 1 ILCs to obesity-associated insulin resistance do not currently exist, and current flow cytometry-based strategies to identify human ILC1s are not specific [9]. However, these results collectively suggest that each member of the group 1 ILCs is sufficient to polarize adipose proinflammatory macrophages through HFD-induced IFN-γ production, and therefore represent a functional spectrum of cells able to contribute to insulin resistance during diet-induced obesity. Other recently proposed mechanisms of how group 1 ILCs increase adipose proinflammatory macrophages during HFD, such as increased TNF-α production [34] or decreased killing of adipose M2 macrophages [36] by group 1 ILCs, are likely secondary to enhanced IFN-γ production, because adoptively transferred *Ifng^−/−^* group 1 ILCs from HFD fed mice do not increase the density of proinflammatory macrophages in lymphocyte-deficient mice during HFD [14]. Therefore, it is more likely that these alternative mechanisms can contribute to obesity-associated systemic insulin resistance by other mechanisms that will need further investigation.

The growing consensus in the field is that group 1 ILCs are sufficient and necessary to drive obesity-associated inflammation in the adipose tissue by polarizing adipose proinflammatory macrophages. However, the mechanisms by which group 1 ILCs are activated during HFD remain unclear. Adipose NK cells from obese patients displayed higher NKG2D levels compared to lean individuals [108], and increased expression of NKG2D ligands was observed in adipocytes from the VAT of obese mice compared to lean controls [70]. However, NKG2D-deficient mice did not display reduced insulin resistance, or increased numbers of proinflammatory macrophages, suggesting that NKG2D is not required for this process [70]. A recent study indicated that NK cell production of IFN-γ is stimulated by ligation of the activating receptor NKp46 by unknown ligands present on VAT adipocytes, and that this pathway is responsible for driving early proinflammatory macrophage polarization in the VAT, but not the SAT [35]. Instead, it is well established that IL-12 and STAT4 signaling are critical for NK cells to produce IFN-γ and proliferate following viral infection [109,110] and elevated IL-12 transcripts are found in the adipose tissues of mice soon after HFD feeding [14,111,112]. In support of these findings in mice, clinical studies have observed higher serum levels of IL-12 in obese individuals compared to lean individuals [113,114]. A recent study also demonstrated that IL-12 is induced as early as 3 weeks after HFD administration in the VAT and SAT, and IL-12 signaling is an absolute requirement for driving the proliferation and accumulation of group 1 ILCs in the adipose tissue during diet-induced obesity [14]. Therefore, while the conflicting results regarding NKp46 ligand induced activation of group 1 ILCs during HFD may be dependent on differences in microbiota or the content of experimental HFD used, early mouse and clinical data suggests that IL-12 plays an important role in this process.

## 4. Concluding Remarks

Evidence is now becoming apparent that ILCs can influence and be influenced by host metabolism, and the cellular and molecular mechanisms are just now becoming elucidated. However, many unresolved questions remain regarding ILC immunometabolism. What are the metabolic pathways that are utilized by ILCs to maintain their tissue-residency and turnover? Can ILC3s influence microbial composition to impact host metabolism? What is the role of adipose-resident group 1 ILCs during homeostasis? Future studies will also need to address whether the observed discrepancies observed in ILC2-intrinsic metabolism during inflammation are due to differences in tissue-specific biosynthetic precursors or model-specific activating signals. Despite these questions, studies of host metabolism collectively support that mouse adipose ILC2s regulate insulin sensitivity of the adipose tissue by production of IL-5 and IL-13, whereas group 1 ILCs may play a detrimental role in mammalian obesity through proinflammatory macrophage polarization and promotion of tissue fibrosis. Given the prevalence and alarmingly increasing rate of global obesity, studies further elucidating the mechanisms by which ILCs influence host metabolism may prove to be beneficial for therapeutic use in obesity-associated diseases such as cancer and type 2 diabetes.

## Figures and Tables

**Figure 1:** Metabolic pathways utilized by innate lymphoid cells (ILCs) during homeostasis and activation. (**A**) Naive ILCs are generally thought to be quiescent and largely use metabolic pathways that efficiently metabolize glucose through glycolysis-linked mitochondrial oxidative phosphorylation (OxPhos) to generate energy in the form of adenosine triphosphate (ATP). However, during inflammation, ILCs respond to increased levels of proinflammatory cytokines that cause their activation and concomitant changes in cellular metabolism. (**B**) Activated natural killer (NK) cells respond to heighten levels of the cytokines IL-12, IL-18, and IL-15 through activation of mammalian target of rapamycin (mTOR) signaling, which is associated with an increased rate of glycolysis to meet higher biosynthetic demand by metabolizing glucose into lactate in a process called aerobic glycolysis. Aerobic glycolysis is needed to provide the cell with essential precursors for amino acids, lipids, and nucleotides to fuel effector function and proliferation. (**C**) Following IL-33 stimulation, activated ILC2s can also increase aerobic glycolysis, which is dependent on arginase-1 (*Arg1*) activity to metabolize extracellular l-arginine into ornithine-derived polyamines to fuel increased glycolysis (left panel). Alternatively, ILC2s take up extracellular long-chain fatty acids through an undefined transporter and utilize mitochondrial fatty acid oxidation (FAO) to fuel proliferation and effector function without the need of glucose uptake (right panel) (**D**) In response to IL-1β and IL-23, ILC3s increase both glucose and fatty acid metabolism and display increased mitochondrial oxygen consumption.
